The article "Intracytoplasmic morphologically selected sperm injection versus conventional intracytoplasmic sperm injection: a randomized controlled trial" was retracted in 2017. Reason: lack of ethics approval or compliance.

# Intracytoplasmic morphologically selected sperm injection versus conventional intracytoplasmic sperm injection: a randomized controlled trial

**DOI:** 10.1186/s12958-015-0096-y

**Published:** 2015-08-27

**Authors:** Giovanni Battista La Sala, Alessia Nicoli, Eleonora Fornaciari, Angela Falbo, Ilaria Rondini, Daria Morini, Barbara Valli, Maria Teresa Villani, Stefano Palomba

**Affiliations:** Obstetrics and Gynecology Unit, Arcispedale S. Maria Nuova of Reggio Emilia, IRCCS, Reggio Emilia, Viale Risorgimento 80, 42123 Reggio Emilia, Italy; University of Modena and Reggio Emilia, Via del Pozzo, 71, 41124 Modena, Italy

**Keywords:** Intracytoplasmic sperm injection, ICSI, Intracytoplasmic morphologically selected sperm injection, IMSI, MSOME, RCT

## Abstract

**Background:**

Intracytoplasmic morphologically selected sperm injection (IMSI) is still proposed and employed in the clinical practice to improve the reproductive outcome in infertile couples scheduled for conventional intracytoplasmic sperm injection (cICSI). The aim of the current randomized controlled trial (RCT) was to test the hypothesis that IMSI gives a better live birth delivery rate than cICSI.

**Methods:**

Infertile couples scheduled for their first cICSI cycle for male factor were allocated using a simple randomization procedure. All available biological and clinical data were recorded and analyzed in a triple-blind fashion.

**Results:**

Our final analysis involved the first 121 patients (48 and 73 subjects for IMSI and cICSI arm, respectively) because the trial was stopped prematurely on the advice of the data safety and monitoring Committee because of concerns about IMSI efficacy at the first interim analysis. No significant difference between arms was detected in rates of clinical pregnancy per embryo transferred [11/34 (32.3 %) *vs.* 15/64 (23.4 %); odds ratio (OR) 1.56, 95 % (confidence interval) CI 0.62–3.93, *P* = 0.343] and of live birth delivery [9/48 (18.8 %) *vs.* 11/73 (15.1 %); OR 1.30, 95%CI 0.49–3.42, *P* = 0.594).

**Conclusion:**

Current data did not support the routine use of IMSI in the clinical practice for improving cICSI results in unselected infertile couples with male factor.

## Background

In the assisted reproductive technologies (ARTs), intracytoplasmic sperm injection (ICSI) represents the treatment of choice for couples with male factor infertility and low or absent fertilization rate in previous conventional in vitro fertilization (IVF) cycles [1]. The ICSI outcome depends on several factors, including oocyte quality, patient’s age and the quality of the single spermatozoa selected to be injected into the oocyte. This selection is usually performed under an inverted microscope with magnification of 200×-400×, that allows to detect both motility and normal morphology of spermatozoa, based on evaluation of their head, neck and tail. However, this selection revealed many limitations because of the low magnification used, that permits to observe only major sperm morphological defects [2].

In order to improve the sperm selection, a new method of human spermatozoa evaluation called “motile sperm organelle morphology examination” (MSOME) was suggested [3]. MSOME allows spermatozoa examination at high magnification (6000× and over) permitting a better morphological evaluation of acrosome, post-acrosomal lamina, neck, tail, nucleus, mitochondria [3] and, thus, the selection of motile spermatozoa with a morphologically normal nucleus, normal nuclear content and mitochondrial function [4–6]. The integration of MSOME method into ICSI procedure led to intracytoplasmic morphologically selected sperm injection (IMSI) [7].

Since the introduction of IMSI twelve years ago, many studies were published comparing the efficacy of IMSI respect to cICSI, with conflicting results. That controversial data may be due to the different studies’ design (comparative, prospective comparative and prospective randomized studies), the application of heterogeneous inclusion criteria (maternal age, previous failed ICSI cycles, ovarian response and number of retrieved oocytes, etc.), and different systems of high magnification sperm morphology classification adopted [8].

A systematic review with meta-analysis [9] aimed to compare IMSI with conventional ICSI (cICSI) in couples with previous cICSI failures or male factor infertility demonstrated improved reproductive outcomes in infertile couples whom received IMSI. Specifically, in couples with previous cICSI failures an implantation rate about three-fold higher [odd ratio (OR) 2.88, 95 % confidence interval (CI) 2.13–3.89], a pregnancy rate two-fold improved (OR 2.07, 95%CI 1.22–3.50) and a miscarriage rate reduced of about 70 % (OR 0.31, 95%CI 0.14–0.67) was observed after IMSI when compared with cICSI [9]. However, although less evident, the data synthesis demonstrated a benefit of IMSI over cICSI also in unselected infertile couple with only male factor [9]. In fact, the implantation (OR 1.56, CI 1.11–2.18) and pregnancy (OR 1.61, 95%CI 1.17–2.23) rates resulted improved by 50 and 60 %, respectively [9].

Moreover, only few studies comparing the efficacy of IMSI versus cICSI in a randomized controlled fashion are available, and with conflicting results [4, 9]. A meta-analysis [10] of randomized controlled trials (RCTs) concluded that the current evidence does not support the clinical use of IMSI since there is no effect on live birth or miscarriage rate, and that the quality of the scientific evidence for a beneficial effect on the clinical pregnancy rate is of very low quality.

Notwithstanding that conclusion, increasingly patients still require an IMSI procedure in case of male factor at their first IVF cycle in order to optimize their reproductive results. Based on these considerations, the current pragmatic RCT was aimed to test the hypothesis that IMSI gives better reproductive results than cICSI in infertile couples scheduled for their first IVF cycle.

## Methods

The present study follows the Consolidated Standards of Reporting Trials (CONSORT) guidelines and their extension for nonpharmacological trials [11, 12]. A further paper’ revision was performed according to the recent guidelines for infertility trials [13]. All terms employed followed the International Committee for Monitoring Assisted Reproductive Technology (ICMART) and the World Health Organization (WHO) revised glossary on ART terminology [14].

### Protocol

The current study was a single-center triple-blind randomized trial. Specifically, the patients’ enrollment study was performed from May 2011 to September 2012 at the Infertility Centre of the ASMN – IRCCS of Reggio Emilia (Italy). The Infertility Centre of Reggio Emilia is a high-volume IVF Unit where about 1,500 IVF procedures are performed yearly.

The Local Ethical Committee approval was not required because the procedure was commonly employed in the clinical practice. All couples (female and male partners) signed an informed consent before the screening procedures for enrolment. At study design, the trial was not recorded on any international register available online. Thus, an international registration number is not actually available.

After patients’ selection according to inclusion and exclusion criteria, a case history was collected for each (male and female) patient, all female patients underwent anthropometric measurements, clinical evaluation, and pelvic ultrasonography. After ovarian stimulation and oocyte retrieval, each infertile couple was randomized to receive in a blinded fashion or standard (i.e., cICSI) or experimental (i.e., IMSI) IVF procedure. All clinical (including safety data and compliance with the treatments) and biological data were recorded by a researcher blinded to patients’ allocation. Pregnancies were followed with a standardized protocol according to National guidelines [15] by the same team of obstetricians who did not know which treatment the patients had received. Obstetrical/neonatal data, as well as all pregnancy complications, were carefully recorded [13]. A follow-up of the offspring was planned at one year of age to assess the health of babies (and to assess congenital abnormalities, long-term effect of pregnancy complications, developmental delays, and so on) [13].

All procedures, drugs, culture media, instruments and visits performed and used during the study were defined at study design and were the same for each couple. It was planned that all oocytes pick-ups and embryo transfers should be performed by the same operator (GBLS).

### Study population

Eligible participants were all couples scheduled to their first ICSI cycle for male infertility with ejaculated fresh sperm. However, the decision of whether to perform IVF or ICSI was definitively made upon sperm quality analysis performed after oocyte pick-up. Specifically, a percentage of spermatozoa with normal morphology less than 4 % [20] and/or a number of activated spermatozoa 1.5 10^6^/ml after capacitation were considered inclusion criteria. A concentration of activated motile sperm less than 0.1×10^6^/mL after swim-up technique, and the use of cryopreserved or surgically retrieved semen were considered exclusion criteria. No other specific exclusion criteria (including a female age > 40 years) was used.

### Randomization

Eligible participants were allocated randomly to two independent arms (cICSI and IMSI arm) using a simple randomization procedure [16]. Specifically, couples were allocated to one of two groups according to the last number of numeric code of the female partner’s identity document (e.g. even-ICSI group and odd-IMSI group). To simplify the blinding procedures, the randomization was performed in the laboratory just before the ICSI procedure. The modality of the randomization was known only to the physician who performed the initial selection and recruitment of couples and was kept hidden from the team for the entire duration of the study. The resulted block size was variable. The random allocations were concealed in closed dark envelope until the end of the study.

All clinicians, investigators, assessors, and patients remained blinded to the treatment assigned until the end of the study. Data analysis was also performed by a researcher who did not know couples’ allocation (triple-blind).

### Interventions

#### Controlled ovarian stimulation and oocyte retrieval

Controlled ovarian stimulation protocols and oocyte retrieval are described elsewhere [17]. Briefly, after ovarian down regulation, obtained with a long luteal leuprolide acetate depot protocol (Enantone 3.75 mg; Takeda, Milan, Italy), recombinant follicle-stimulating hormone (rFSH; Gonal F; Serono, Rome, Italy) was administrated using a starting dose (first five days) tailored according to patient’s age and antral follicle count (ranged from 112.5–450 IU/day). From day 6 of ovarian stimulation, the ovarian response was monitored by transvaginal ultrasonography and serum estradiol (E_2_) assay every 3 days up to the appearance of dominant follicles with a mean diameter of at least 12 mm and, then, daily. The dose of rFSH was adjusted according to the ovarian response. When one or more > 17 mm in diameter were obtained, the ovulation was triggered by injection of 10,000 IU human chorionic gonadotropin (hCG) 24 h after the last injection of rFSH, and 36 h later oocyte retrieval was performed by ultrasound-guided transvaginal aspiration. The cycle was canceled in patients at high risk for ovarian hyperstimulation syndrome (OHSS) [18], whereas a low ovarian response was not considered an indication to cancel the cycle.

#### Semen preparation, sperm selection and oocyte injection

Semen samples were collected by masturbation after 3–5 days of ejaculatory abstinence and evaluated according to the threshold values established by last WHO manual [19]. Sperm morphology was evaluated according to strict Kruger criteria [20]. Semen preparation was performed as previously described [17]. Briefly, after liquefaction semen sample was diluted with 10 mL of buffer medium (G-MOPS Plus; Vitrolife, Gothenburg, Sweden) and centrifuged 10 min at 800× g at room temperature. After supernatant removal, the pellet was diluted with 5 mL of buffer medium and centrifuged 10 min at 800× g at room temperature. The supernatant was removed and the pellet was overlaid with 1 mL of medium (G-IVF Plus; Vitrolife, Gothenburg, Sweden) and incubated at 37 °C, 6 % CO_2_ in air to separate by swim up. In case of semen with sperm concentration < 1 × 10^6^/mL, the sample was concentrated by one centrifugation at 1500× g and the pellet removed in 1 mL of medium.

cICSI procedure was performed 3 h after the oocyte retrieval in a plastic dish of 50 mm × 9 mm (Ref. 351006; BD Biosciences Labware, Belgium) with 5 μl microdroplets (G-MOPS Plus; Vitrolife, Gothenburg, Sweden) for oocyte injection and a droplet of polyvinylpyrrolidone droplet (PVP; Vitrolife, Gothenburg, Sweden) covered with mineral oil (Ovoil; Vitrolife, Gothenburg, Sweden). An aliquot of sperm suspension was added to PVP for the search and capture of spermatozoa selected for injection.

cICSI was performed with an inverted microscope (TE 2000 U; Nikon Corp., Tokyo, Japan) equipped with a heated stage (37 °C) and the Hoffman modulation contrast under ×200 magnification [21]. In case of cICSI, the embryologist excluded spermatozoa exhibiting severe morphological defects with particular regard for the head.

All IMSI procedures were always performed by only one experienced and trained operator (BV) in order to limit the inter-operator variability of selection. IMSI started 1 h after the oocyte retrieval and was performed at room temperature with the same inverted microscope (TE 2000 U, Nikon Corp., Tokyo, Japan) equipped with Normarski optics (×60) enhanced by a videozoom, and digital imaging was used to obtain a magnification of ×7000. Firstly, an aliquot of sperm suspension was added to a PVP droplet (PVP; Vitrolife, Gothenburg, Sweden) covered with mineral oil (Ovoil; Vitrolife, Gothenburg, Sweden) within a glass-bottomed dish (Will Co. Dish® Gwst 5040, Amsterdam, The Netherlands). The evaluation and capture of the spermatozoa was performed as described by Bartoov *et al.* [7, 22], that defined as a “normal” the spermatozoa nuclei with normal-shaped, smooth, symmetric, with oval configuration, and with nuclei presenting a homogeneous nuclear chromatin mass, without regional nuclear disorders and containing no more than one vacuole which occupies less than 4 % of the nuclear area.

No adjustment of the sample temperature and the PVP concentration was made [23]. Moreover, considering data showing a deleterious effect of the sperm manipulation after 2 h [24], it was planned that, if no spermatozoa with normal nuclei were available, the “second best” and the “third best” morphologically evaluated spermatozoa would be retrieved after the first 60 min and 75 min, respectively, hour in order not to complete the sperm collection for IMSI procedures within 1 h and 30 min. In this case, the spermatozoa captured could present a small or large oval nuclear shape with morphologically normal nuclear content (first choice), a non-oval, abnormal nuclear shapes but with normal nuclear content (second choice) or a regional shape disorder (third choice) [25]. Sperm cells exhibiting large nuclear vacuoles but with normal oval nuclear shape were considered preferable for selection to those with combined nuclear malformations [25]. Before the injection, the selected sperm were immobilized and incubated for 30 min (at 37 °C, 6 % CO_2_).

For cICSI and IMSI procedures, the oocytes were denudated and the metaphase II (MII) oocytes were injected within 3 h from oocyte retrieval. Then, the injected oocytes were transferred into 30 μL droplets of culture medium (G1; Vitrolife, Gothenburg, Sweden), covered with mineral oil (Ovoil; Vitrolife, Gothenburg, Sweden) and incubated at 37 °C (6 % CO_2_ in air).

#### Fertilization, embryo cleavage and embryo quality assessment

Oocyte fertilization was assessed 18–20 h after injection [17]. Embryo cleavage and quality were evaluated 48–72 h after injection. For each embryo we evaluated the following parameters: number and regularity of blastomeres (shape and dimension), percentage of fragmentation, appearance of the cytoplasm, symmetry of cleavage and presence and numbers of nuclei [26]. Specifically, embryos characterized by blastomeres having regular shape and dimension, absence of fragmentation and homogeneous cytoplasm without vacuoles and granulation were classified as grade I and considered top-quality embryos; embryos characterized by regular or slightly irregular shape and/or dimension of blastomeres, absence of fragmentation and homogeneous cytoplasm with no more than 10 % of fragmentation as grade II; embryos characterized by irregular shape and/or dimension of blastomeres, fragmentation variable between 10 –30 % as grade III; and embryos characterized by irregular shape and/or dimension of blastomeres, cytoplasmic fragmentation between 30 –50 %, blastomeres with dark or granulose cytoplasm or with numerous vacuole as grade IV; embryos characterized by indistinguishable or degenerated blastomeres, more than 50 % of fragmentation, very dark cytoplasm or high vacuolation or non-developing embryos as grade V [26].

#### Embryo transfer

Embryo transfer was performed 48–72 h after insemination at stage of 4–8 cells by the same operator (GBLS). The number of cleavage embryos to transfer was established according to our internal guidelines based on female age and semen quality. Specifically, in patients with female age < 38, 38–39 and 40–42 years old were transferred 2, 3 and 5 embryos, respectively. In case of sperm concentration < 1 × 10^6^/mL, in patients with <38 and 38–42 years old were transferred 3 and 5 embryos, respectively. All supernumerary embryos, as well as those of patients at risk for OHSS, were cryopreserved, and transferred two cycles later in case of first IVF failure.

All patients undergoing embryo transfer received supplemental progesterone vaginally (400 mg/day for 15 days; Prometrium, Rottapharm, Milan, Italy).

### Main outcome measures

The primary endpoint of the current clinical trial was the live birth delivery rate. The secondary endpoints were the rates of total live birth delivery, healthy baby-in-arm, clinical pregnancy rate, as well as the fertilization rate, the good quality embryos rate, the implantation and the miscarriage rates. Other secondary endpoints were the OHSS and multiple pregnancy rates, the incidence of pregnancy complications, the rate of compliant patients who repeated the IVF procedure after failure.

The live birth delivery rate was defined as the number of deliveries that resulted in at least one live born expressed per initiated (patient), aspirated and embryo transfer cycles [14]. The total live birth delivery rate was defined as the number of deliveries that resulted in at least one live born expressed per 100 couples including all fresh cycles and all frozen/thawed ART cycles [14]. The total healthy baby-in-arm rate was arbitrary defined as the number of healthy babies at one-year follow-up per 100 couples (including all ART cycles per patient). The clinical pregnancy rate was defined as the number of clinical pregnancies expressed per 100 initiated, aspirated and embryo transfer cycles [14].

Pregnancy was initially determined 12 days after embryo transfer by a positive quantitative serum βHCG assay > 10 IU, followed by another quantitative βHCG after 2–4 days to ensure the appropriately rising levels or to confirm the negative result. Clinical pregnancy was defined as at least one fetus with a positive heart beat revealed by transvaginal sonography 4 or 5 weeks after embryo transfer [14].

Fertilization rate was expressed as the number of 2PN zygotes obtained divided by the number of inseminated oocytes; the percentage of good quality embryos obtained was expressed as the number of good quality embryos obtained divided by the total number of embryo obtained; the implantation rate was defined as the number of gestational sacs observed divided by the number of embryos transferred; the miscarriage rate was expressed as the number of miscarriage occurred before 20 weeks of gestational age divided by the number of clinical pregnancies [14].

Other secondary endpoints regarded the pregnancy/maternal and perinatal/neonatal outcomes. Specifically, for each pregnant women were recorded the weight gain, the pregnancy complications (pregnancy-induced hypertension, pre-eclampsia, gestational diabetes mellitus, and so on), the mode of delivery, and the intrapartum complications (hemorrhagia, shoulder dystocia, and so on). For each born, the following data were noted: gestational age at delivery, birth weight, neonatal growth, sillbirth or neonatal death, Apgar score, admission to neonatal intensive care unit, perinatal/neonatal complications (respiratory distress syndrome, hypoglycemia, hyperbilirubinemia, and so on), breastfeeding and its duration. At one follow-up, for each baby a neonatologist searched/excluded anatomic anomalies, neurological deficits, and any generic neonatal disease.

### Statistical analysis

The goal of the proposed superiority study was to test the null hypothesis that in infertile couples with male factor the live birth delivery rate is higher after IMSI than after cICSI. The criterion for significance (alpha error) was set at 0.05. The test was two-tailed, which meant that an effect in either direction would be interpreted. Considering previous RCT showing live birth data [27], the rates of live births for patients undergoing IMSI and cICSI procedure were approximately 0.44 and 0.38, respectively. Thus, we needed to enroll at least 179 patients in each arm to yield a statistically significant result with a power (beta error) of 80 %. To allow for an unpredictable number of withdrawals, we decided to enroll a total of at least 200 patients per arm in the expectation that at least 179 patients would remain. At study design, interim analyses were planned (one every five months) in order to monitor the safety of the experimental procedure and recalculate the sample size. The power analysis and the calculation of sample size were performed using SamplePower, release 2.0.

Data were analyzed using the intention-to-treat (ITT) method on the basis of the treatment assignment. The normal distribution of continuous variables was evaluated using the Kolmogrov-Smirnov test. Continuous data were expressed as the mean ± standard deviation (SD) or as median and interquartile range (IQR) with min-max values. Difference between arms were analyzed by Student *t* test for unpaired data or with Mann–Whitney *U* test, as appropriate. For categorical variables, the Pearson Chi square test was performed; Fisher’s exact test was used for the frequency tables when more than 20 % of the expected values were lower than five.

Cox proportional-hazards model was used to calculate the OR and its 95 % CI for the most relevant clinical endpoints (StatsDirect, release 2.4.3). The number need to treat (NNT) was calculated for the primary endpoint. The level of statistical significance was set at *P* < 0.05 for all statistical analyses. The Statistics Package for Social Sciences (SPSS 15.0.1, 22 November 2006; SPSS Inc., Chicago, IL, USA) was used for all calculations.

## Results

In Fig. 1 is showed the study flow-chart according to the CONSORT guidelines [12, 13]. The patients’ enrolment was stopped prematurely in September 2012 on the advice of the data safety and monitoring Committee because of concerns about IMSI efficacy at the third interim analysis. In fact, a significant and unexpected lower fertilization rate was observed in IMSI arm when compared to cICSI arm. Thus, our final analysis involved the first 121 patients (73 and 48 subjects for cICSI and IMSI arm, respectively) who had been enrolled and randomized. Moreover, pregnant patients were followed up to June 2013 and the follow-up of the offspring was closed in July 2014.

**Fig. 1:** Trial flow-chart according to the CONSORT guidelines [12, 13]

As showed in Table 1 the IMSI and cICSI groups were similar in terms of male and female ages. There was no difference between the two arms also in terms of body mass index (BMI), stimulation length, gonadotropins dose administered, number of dominant follicles and peak of E_2_ levels on day of ovulation triggering (Table 1). The rate of patients with severe male factor (sperm count <1×10^6^/mL) was also not significantly different between two groups [9/73 (12.3 %) and 6/48 (12.5 %) subjects for cICSI and IMSI arm, respectively; *P* = 1.000].

**Table 1:** Clinical characteristics of two study arms

	IMSI	cICSI	*P*
Number of couples	48	73	-
Female age	35.4 ± 4.2	36.1 ± 4.1	0.365
Male age	39.3 ± 6.0	37.7 ± 6.0	0.154
Female BMI	22.9 ± 3.4	23.4 ± 4.5	0.513
Duration of the infertility (mo)	19.5 ± 5.1	18.2 ± 3.9	0.116
Primary infertility (n.; %)	44/48; 91.7	70/73; 95.9	0.434
Co-causes of infertility			
Oligo-anovulation (n.; %)	12/48; 25.0	16/73; 21.9	0.826
Tubal factor (n.; %)^a^	4/48; 8.3	6/73; 8.2	1.00
Stimulation length (days)	12.9 ± 4.0	13.2 ± 3.3	0.654
Gonadotropins dose (IU)	2169.9 ± 1077.5	2536.8 ± 1534.1	0.153
Dominant follicles on day of ovulation triggering (n.)	5.6 ± 2.6	4.9 ± 2.7	0.160
Peak of E_2_ levels on day of ovulation triggering (pg/mL)	1356.3 ± 724.8	1255.0 ± 720.6	0.453

Data expressed as mean ± SD. *BMI*: body mass index. ^a^in no case unilateral/bilateral hydrosalpinges was detected at ultrasonography

No statistically significant differences between IMSI and cICSI arms in terms of baseline semen parameters, and number of retrieved oocytes, number of MII retrieved oocytes and number of inseminated oocytes was observed (Table 2). In 160/219 (73.0 %) spermatozoa with normal nuclei were used for IMSI. In 33/219 (15.1 %), 21/219 (9.6 %) and 5/219 (2.3 %) of cases, the first, the second and the third choice spermatozoa selected were used for IMSI (Table 2). Only in four cases [4/48; (8.3 %)] no spermatozoa with normal nuclei were available for microinjection in IMSI group.

**Table 2:** Biological and clinical outcomes of two study arms

	IMSI (n. 48)	cICSI (n. 73)	*P*
Sperm count (million/ml)	22.6 ± 24.6	22.9 ± 23.7	0.947
Motility (% total count)	29.6 ± 16.0	24.5 ± 12.8	0.055
Morphologically normal spermatozoa (% total count)	2.9 ± 2.2	2.8 ± 2.3	0.812
Sperm morphology by MSOME criteria (n., %)			
Normal nuclei	160/219; 73.0	---	---
First choice selected sperm	33/219; 15.1	---	---
Second choice selected sperm	21/219; 9.6	---	---
Third choice selected sperm	5/219; 2.3	---	---
Aspirated cycles (n.)	48	73	---
Retrieved oocytes (n.)	6.3 ± 2.7	6 ± 3.5	0.6157
MII oocytes retrieved (n.)	5.1 ± 2.5	5.3 ± 3.1	0.709
Oocytes inseminated (n.)	4.6 ± 1.9	4.6 ± 2.8	1.000
Fertilization rate (n.; %)	105/219; 47.9	211/333; 63.4	0.001
Embryo obtained (n.)	99, 2.1 ± 1.7	221, 3.0 ± 1.9	0.009
Good quality embryos rate (n.; %)	73/99; 73.7	167/221; 75.6	0.834
ET rate (n.; %)	34/48; 70.8	64/73; 87.7	0.038
Embryo transferred (n.)	65, 1.4 ± 1.0	137, 1.9 ± 1.2	0.018
Implantation rate (n.; %)	15/65; 23.1	18/137; 13.1	0.102
Total pregnancies (n.)	14	19	---
Total pregnancy rate//initiated cycles (n.; %)^a^	14/48; 29.2	19/73; 26.0	0.865
Total pregnancy rate/ET (n.; %)	14/34; 41.2	19/64; 29.7	0.952
OHSS rate (n.; %)	5/48; 10.4	6/73; 8.2	0.930
Biochemical pregnancy rate (n., %)	3/14; 21.4	4/19; 21.1	0.859
Clinical pregnancies (n.)	11	15	---
Clinical pregnancy rate/initiated cycles (n.; %)*	11/48; 22.9	15/73; 20.5	0.823
Clinical pregnancy rate/ET rate (n.; %)	11/34; 32.3	15/64; 23.4	0.349
Miscarriage rate (n.; %)	2/11; 18.2	4/15; 26.7	1.000
Multiple pregnancies rate (n.; %)	4/11; 36.4	4/15; 26.7	0.683
Delivery live births (n.)	9	11	---
Delivery live birth rate/initiated cycles (n.; %)*	9/48; 18.8	11/73; 15.1	0.624
Delivery live birth rate/ET (n.; %)	9/34; 26.5	11/64; 17.2	0.301
Twin deliveries	2/9; 22.2	4/11; 36.4	0.496
Live births	11	14	
Cycles with embryo freezing	9/48; 18.8	13/73; 17.8	0.895
Embryo thawing cycles	9	7	----
Embryo thawing ET	6/9; 66.7	5/7; 71.4	0.839
Embryo thawing clinical pregnancies	0/6; 0	2/5; 40	0.186
Embryo thawing deliveries	0/6	1/5; 20	0.528
Total delivery live birth rate/initiated cycle (n., %)	9/48; 18.8	12/73; 16.4	0.743

Data expressed as mean ± SD or as number/percentage. *MII* metaphase II, *MOSOME* motile sperm organelle morphology examination, *PU* pick-up, *ET* embryo transfer, *OHSS* ovarian hyperstimulation syndrome, ^a^Because no cycle was cancelled, the initialled cycles corresponded to the aspirated cycles

The fertilization rate, as well as the number of embryos obtained, number of embryo transfers performed and the mean number of embryos transferred, were significantly higher in the ICSI arm. The percentage of good quality embryos obtained was similar in the two study arms (Table 2).

No significant difference between study arms was detected in any of the other main outcome measures; specifically, the delivery live birth rates per initiated cycles [9/48 (18.8 %) *vs.* 11/73 (15.1 %) for IMSI and cICSI arms, respectively; *P* = 0.624] and per embryo transfer [9/34 (26.5 %) *vs.* 11/64 (17.2 %) for IMSI and cICSI arms, respectively; *P* = 0.301] were not significantly different (Table 2). The ORs for the delivery live birth rates per initiated cycles and per embryo transfer were 1.30 (95 % CI 0.49 to 3.42, *P* = 0.594), and 1.73 (95 % CI 0.64–4.62, *P* = 0.281; respectively. The NNT for IMSI procedure was of 28 benefits. Reproductive data after inclusion of frozen IVF cycles did not change significantly our findings (Table 2). No effect of the specific IVF procedure used was detected on further fertility treatments [43/48 (89.6 %) *vs.* 56/73 (76.7 %) for IMSI and cICSI arms, respectively; *P* = 0.093].

Obstetrical e neonatal data were not significantly different between the two study arms (Table 3).

**Table 3:** Obstetrical e neonatal data in the two study arms

	IMSI (n. 48)	cICSI (n. 73)	*P*
Maternal outcomes			
Pregnancy complications (n.; %)	4/9; 44.44	1/12; 8.33	0.080
Mode of delivery			
Spontaneous delivery (n.; %)	5/9; 55.55	6/12; 50	0.801
Instrumental delivery (n.; %)	1/9; 11.11	1/12; 41.67	0.831
Caesarean delivery (n.; %)	3/9; 33.33	5/12; 36.36	0.698
Intrapartum complications (n.; %)	1/9, 11.11	1/12, 9.09	0.831
Neonatal outcomes			
Gestational age at delivery (weeks)	36.25 ± 2.77	38.03 ± 1.58	0.077
Preterm delivery (n.; %)	2/9, 22.2	2/12, 16.7	0.749
Birth weight (g)	2535.00 ± 710.00	2789.37 ± 575.24	0.492
Apgar score at 5 min	8.80 ± 0.45	9.33 ± 0.82	0.211
Admission to NICU (n.; %)	2/11; 18.18	1/15; 7.14	0.382
Breastfed babies (n.; %)	1/11; 9.09	1/15; 7.14	0.819
Duration of breastfeeding (months)	6.33 ± 5.13	6.6 ± 5.08	0.906
Congenital anomalies (n.; %)	2/11; 18.18	0	0.190

Data expressed as mean ± SD or as number/percentage. *NICU* neonatal intensive care unit

All biological and clinical data obtained resulted not influenced by severe male factor infertility, different operator (for cICSI) and patient’s BMI (data not shown).

## Discussion

The purpose of this RCT was to verify in our clinical practice the impact of the use of IMSI in couples who attempted at their first ICSI cycle for male factor. In this view, only couples with sperm concentration less than 0.1×10^6^/ml after semen preparation were excluded from this study in order to have a sufficient number of spermatozoa to perform an effective selection, whereas no specific criteria was used for selecting female subjects. Obviously, in our study population a consistent proportion of patients was aged more than 38 years and/or poor responders. This translated with a low reproductive performance in both arms with particular regard for the rates of fertilization.

Our data demonstrated that IMSI procedure did not improve the reproductive outcomes in infertile couples scheduled for cICSI. In particular, no significant difference was detected for live birth delivery rate, our primary endpoint. Current results confirm those obtained in two previous RCTs on unselected populations of infertile couples [27, 28]. Moreover, the Leandri’s study [28] had a multicenter design with a number of biases and confounders [11], and included only female patients younger than 39 years and day 3 FSH level lower than 9 IU/L. The data synthesis of these two studies [27, 28] with the current demonstrates no clinical benefit of IMSI over cICSI (Fig. 2). Specifically, IMSI resulted in a significantly higher rates of implantation (OR 1.40, CI95% 1.06–1.88, *P* = 0.02) with moderate heterogeneity (*I*^*2*^ = 33 %) but no significant difference in terms of clinical pregnancy rates and, most important, live birth rates was observed (OR 1.12, 95 % CI 0.78–1.61, *P* = 0.53 with *I*^*2*^ = 0 % and OR 1.04, 95 % CI 0.72–1.52, *P* = 0.83 with *I*^*2*^ = 0 %; respectively).

**Fig. 2:** Data synthesis for the main reproductive outcome measures of the published RCTs on unselected infertile populations

Although in the current trial no effect on all biological and clinical data was detected by severe male factor infertility, at the moment, it cannot exclude that IMSI could have a beneficial effect in selected couples. After data sub-analysis, Balaban *et al. *[27] demonstrated an higher implantation rate after IMSI in couples with severe male factor infertility suggesting that the IMSI technique could exert some benefit for selected couples. In the first RCT published by Antinori and co-workers, IMSI significantly increased the implantation and the clinical pregnancy rates, particularly in couples with two or more cICSI failures [29]. Other recent non-randomized studies demonstrated that IMSI could improve clinical outcomes in couples with teratozoospermia [30, 31], even if no benefit of IMSI in infertile couples with isolated male factor and at least six oocytes available on retrieval was demonstrated in a RCT [32]. In fact, the absolute difference in clinical pregnancy rate between IMSI and cICSI was less than 1 % (36.8 % *vs.*37.2 %, respectively) [32]. After data subanalysis, better results were obtained in patients with oligoasthenoteratozoospermia defined according to 2010 WHO references values [32]. However, those results were not obtained in a randomized populations resulting potentially biased by several confounders [32]. Finally, more recently, IMSI was also studied in couples with women with poor ovarian response to gonadotropin stimulation [33] or with advanced age [6]. In particular, poor responders did not benefit from sperm selection under high magnification prior to ICSI [33], whereas IMSI resulted in an improved embryo quality and in a 9-fold increase in the clinical pregnancy rate in selected couples with advanced maternal age and good ovarian response [23].

Overall, our data show slight differences between cICSI and IMSI in terms of biological result, such as the fertilization rate, the number of embryos obtained, number of embryo transfers performed and the mean number of embryos transferred. These results do not depend on differences in semen and oocytes characteristics, as well as in the percentage of couples with severe male factor infertility. An effect of morphology of spermatozoa selected for IMSI can be excluded. In fact, only in few cases were not available spermatozoa with normal nuclei for microinjection. An effect of the time can be excluded too. In fact, all IMSI procedures were completed within 90 min, as defined in the study protocol. The risk for a damage of the sperm membrane due to PVP exposure [34] was minimized in our study. Notwithstanding we limited the time of sperm selection, in a very high proportion of cases the “best” one spermatozoa was injected. To this regard, it is well known that the injection of spermatozoa with morphological defects significantly reduces the fertilization rate, the percentage of top-quality embryos obtained, the implantation and the clinical pregnancy rates [25, 35].

A significant effort was to assess the impact of IMSI procedure on other ancillary secondary endpoint. Firstly, no beneficial or worsening impact of the IMSI can be suspected on the compliance of the couples to further fertility treatments. Secondly, no effect of IMSI was observed on the incidence of obstetric complications and on pregnancy outcome, including maternal and neonatal/fetal outcomes. Moreover, our data cannot exclude higher (or lower) birth defects and epigenetic diseases. To this regard, only one peer-reviewed study was published on the incidence of major congenital malformation of 1028 children born after IMSI or cICSI [36]. A reduced risk for major birth defects was observed after IMSI, also after multivariate adjustment for confounding factors [36]. That result confirmed a preliminary non-peer-reviewed report on a small sample, not published further in extension [37].

Current RCT has specific strengths and limitations. The strengths regard the study design, setting care given, and the lack of patients’ selection. It had a prospective randomized design with patients blinded to the procedure received and assessors blinded to the patients’ allocation. The setting was a high-volume center for IVF procedures, and the biologists were specifically trained and certified for both procedures. Our primary endpoint was the live birth rate, albeit a one-year follow-up was initially planned to confirm the health of the babies born [13]. In addition, our study was performed on unselected couples at their first IVF cycle. In fact, according to the definition of pragmatic trial, in our opinion the use of no specific exclusion criteria for female partner must be considered a study’ strength since our sample was totally representative of population of couples referring for an IVF cycle for male infertility. Moreover, our study had also limitations essentially due to little sample size and the unbalanced number of patients allocated in the IMSI and cICSI groups. In fact, the current clinical trial was prematurely stopped at the first interim analysis. The need to stop a study protocol after negative data on intermediate endpoints can be issue of discussion. However, this induced a loose of study’ power and accuracy to drawn definitive conclusions. In addition, it could have reduced the effect of randomization in reducing the selection bias balancing the arms with respect to many known and unknown confounding or prognostic variables. Furthermore, the simple randomization seemed to be still effective since the two study arms resulted homogeneous for all clinical and biological parameters assessed and any statistical correction was need.

## Conclusion

Current data suggests that IMSI did not improve any reproductive outcome in unselected infertile couples scheduled at their first cICSI cycle. Thus, at the moment, it is not justifiable introducing IMSI in the clinical practice and that procedure should be performed only in a research setting with the aim to clarify its real efficacy in well selected populations.

## Abbreviations

ART: Assisted reproductive technologies
BMI: Body mass index
CI: Confidence interval
cICSI: conventional ICSI
CONSORT: Consolidated Standards of Reporting Trials
E_2_: Estradiol
hCG: Human chorionic gonadotropin
ICMART: International Committee for Monitoring Assisted Reproductive Technology
ICSI: Intracytoplasmic sperm injection
IMSI: Intracytoplasmic morphologically selected sperm injection
IVF: In vitro fertilization
MSOME: Motile sperm organelle morphology examination
NNT: Number need to treat
OHSS: Ovarian hyperstimulation syndrome
OR: Odds ratio
PVP: Polyvinylpyrrolidone
RCT: Randomized controlled trial
rFSH: Recombinant follicle-stimulating hormone
WHO: World Health Organization
